# Evaluation of Behavior of 13X Zeolite Modified with Transition Metals for Catalytic Applications

**DOI:** 10.1155/2022/7352074

**Published:** 2022-10-26

**Authors:** Elena. David

**Affiliations:** National Research Institute for Cryogenic and Isotopic Technologies, Street Uzinei No. 4, P. O Raureni P.O. Box 7, 240050 Ramnicu Vâlcea, Romania

## Abstract

This work was intended to develop catalysts based on 13X zeolite modified with transition metals for catalytic applications. In this regard, 13X zeolite was modified by loading of transition metals such as Fe, Co, Cu and various types of catalysts such as Fe-, Co-, Cu-, Fe-Co-, Fe-Cu-, and Co-Cu/13X zeolite were obtained. To prepare these catalysts, the wet impregnation method and metallic precursors were used. The catalysts were characterized by SEM, XRD, BET, and ammonia adsorption. Then the catalytic performance was investigated during upgrading of rapeseed residual biomass pyrolysis vapors using this catalysts and a fixed-bed reactor in two stages. Experimental results showed that the addition of transition metals improved the catalytic selectivity towards aromatic hydrocarbons and Fe-Cu/13X zeolite catalyst was the best and had a high deoxygenation activity (from 62.45% to 20.56%), produced maximum monoaromatic hydrocarbons (of 27.45%), the oxygen content in bio-oil was reduced from 34.98 wt% to 16.06 wt%, the calorific value increased and thus the bio-oil quality was improved.

## 1. Introduction

Energy demand has grown rapidly in recent years due to industrial development and population needs, leading to intense exploitation and massive consumption of fossil fuels [1]. The use of large amounts of fossil fuels has led to the release into the atmosphere of huge volumes of greenhouse gases (GHG) that cause global warming and unwanted climate change [2]. As biomass is a renewable and carbon-neutral source of raw material, it can be a potential and alternative source of energy due to its spread throughout the world, abundance, inexpensiveness, and regenerative properties [3–5].

For the conversion of biomass into energy and value-added chemicals, several technologies based on thermochemical and biological processes are being developed [1, 6, 7]. Of these, the technologies based on thermochemical processes such as gasification, pyrolysis, carbonization, and liquefaction are the most used to produce energy from biomass and value-added chemicals. The pyrolysis process is usually used to obtain solid, liquid, and gaseous products from biomass [1, 6, 8]. The liquid fraction obtained as a pyrolysis product is known as bio-oil and is a dark brown liquid that contains oxygenated compounds such as acids, alcohols, phenols, aldehydes, esters, and ketones [9]. Due to this composition, the bio-oil has undesirable properties such as high oxygen and water content, high acidity and viscosity, and low heating value that do not make it possible to use it directly as a fuel or as a fuel additive [10–12].

In order to use bio-oil as a fuel, it is necessary to improve its quality so that the maximum oxygen content is below 3 wt. %, the water content does not exceed 0.2 g/kg, viscosity must be in the range from 2 to 4.5 mm^2^/s, at 40°C, in accordance with the regulations in force [13, 14]. The purpose of the upgrading process of raw pyrolysis bio-oil is to reduce the oxygen content to improve stability, increase the pH to reduce corrosion problems due to low pH, decrease the viscosity for easy pumping in the engine, reducing the problems associated with storage and transport due polymerization reactions, and increase of heating value by increasing the content of monocyclic aromatic hydrocarbons (MAHs) and aliphatic hydrocarbons [15, 16]. In recent years, many studies have been conducted to investigate the introduction of catalysts in the pyrolysis process to obtain products (bio-oil, bio-char, and biogas) with improved quality [15, 17–20]. Also, the literature presents many studies [21–23] regarding the valorization of biomass waste resulting in biofuels and biochemicals production. Aysu and Durak [21] carried out the study to describe the slow pyrolysis of giant mullein (*Verbascum thapsus* L.) stalks in a fixed-bed tubular reactor with (Al_2_O_3_, ZnO) and without catalyst at different temperatures between 400 and 550°C, at a constant heating rate and also a constant stripping gas (N_2_) flow rate. The yields of bio-char, bio-oil, and gas resulted were determined and the compositions of the obtained bio-oils were established using gas chromatography-mass spectrometry. The results showed that both temperature and catalyst have significant effects on the conversion of *Verbascum thapsus* L. biomass into solid, liquid, and gaseous products. Alayont, et al., [22] in their study, presented the pyrolysis of biomass (*Sinapis arvensis*) that first was pretreated with acidic (H_2_SO_4_, HCI) and alkaline (NaOH, KOH) agents and also high temperature water. After pretreatment, these samples were pyrolyzed at different temperatures (350, 450, and 550°C). The products obtained at the end of the pyrolysis process were characterized, and it was found that alkaline and acidic pretreatment increased the liquid fraction yield and also supported the formation of high energy value bio-char. The properties of the bio-oil and bio-char obtained changed according to the pretreatment method used.

In another study, [23] Durak and Aysu describe the slow pyrolysis of avocado seeds (Persea americana) biomass that was performed in a fixed-bed tubular reactor with and without catalyst, at three temperatures ranging from 400 to 600°C, with a heating rate of 50°C/min. The influences of pyrolysis parameters such as temperature and catalysts, on product yields were investigated and it was found both temperature and catalysts are the main factors affecting the conversion of avocado seeds biomass into solid, liquid, and gaseous products.

The pyrolysis process in two stages leaded to significant improvements on the quality of bio-oil, in the first stage, a thermal decomposition takes place and in the second stage the generated vapors in first stage pass through the catalyst bed, where the pyrolysis intermediate compounds are converted to hydrocarbons [24, 25]. The catalysts based on zeolites are commonly used for the upgrading of the bio-oil because of their three-dimensional pore structure, high surface area, shape selectivity, and acid sites. Also, they have a high reactivity for cracking, aromatization, and isomerization reactions, and can selectively convert the compounds containing oxygen to aromatics and aliphatic hydrocarbons [26–28]. All catalysts used in their researches reduced the compounds containing oxygen from the bio-oil composition. Other authors [29, 30] have found that ZSM-5-based catalysts have higher selectivity to produce aromatic hydrocarbons, but in the same time they pointed out that a high amount of polycyclic aromatic hydrocarbons (PAHs) can produce the coke, the effect being in the catalysts deactivation [29]. To solve this problem, metal-modified zeolite catalysts with acid sites and metal sites [18, 27] have been developed and studied. To modify the zeolites, the transition metals were usually used such as Fe, Ni, Cu, Zn, Co, Pd, Ga, Zr, Mo, Mn, and Ce, and the resulted catalysts were employed for the catalytic upgrading of bio-oil [30–32]. The modification of zeolites by the addition of transition metals aims to increase the selectivity to monocyclic aromatic hydrocarbons and reduce the amount of polycyclic aromatic hydrocarbons to reduce the formation of coke on the surface of the catalyst and its deactivation [29]. On the other hand, the properties of 13X zeolite compared with other types of zeolites (for example, ZSM-5 that is known as having a high activity and a good behavior in biomass conversion processes) found that 13X zeolite has a larger specific surface area than ZSM-5, 620 m^2^/g compared to 420 m^2^/g, respectively [33], the average pore diameter of the 13X zeolite is larger than that corresponding to the ZSM-5 zeolite (1 nm compared to 0.54–0.56, respectively) [34], and taking into account that biomass intermediates have larger molecules, 13X zeolite could be a suitable catalytic material for biomass conversion if is modified by adding transition metals into its mass. As mentioned above, many kinds of biomass have been considered as energy crops and rapeseed *(Brassica napus L.)* is one of these crops and it can be cultivated nearly all over the world. Its annual global production is estimated to be several million tonnes, hence, the importance of rapeseed as an energy crop is gradually rising [35]. There are many studies about the investigation of processing of rapeseed by pyrolysis or gasification processes under various conditions. Pyrolytic decomposition investigations were performed under inert conditions to obtain liquid, solid, or gaseous products [36–38]. Gross calorific value of bio-oil produced from rapeseed biomass wastes ranges around 18.5–20.5 MJ/kg [37, 38] and this makes the rapeseed biomass waste to be a suitable source for energy and bio-oil production. However, the bio-oil produced from rapeseed biomass waste still needs further upgrading to improve its quality and also there is lack of data on catalytic pyrolysis of this biomass waste. For these reasons, it is required to further study the catalytic pyrolysis process and to develop new types of catalysts with increased performance. In a number of studies [39–41], commercial and laboratory-synthesized catalysts have been evaluated for their performance in improving the characteristics of pyrolysis bio-oil.

The experimental results showed that the ZSM-5 zeolite modified with iron used as catalyst achieved the high yield of hydrocarbons in bio-oil composition. In another study [42], the catalytic fast pyrolysis of pine sawdust with a series of Mo–Cu/HZSM-5 catalysts was investigated. The obtained results showed that Mo (3%)-Cu (3%)/HZSM-5 produced the high amount of C_6_-C_12_ hydrocarbons, and converted CH_4_ to bio-oil. As a conclusion, if the pyrolysis vapors contain C_1_-C_3_ hydrocarbons, the HZSM-5 zeolite modified with Mo, Cu, Zn, and Fe used as catalysts will increase the aromatic hydrocarbons yields. Due to the similar characteristics, between the ZSM-5 zeolite and the 13X zeolite, it is assumed that the 13X zeolite modified with transition metals can be a catalyst with a good performance and behavior in the upgrading process of the pyrolysis bio-oil. Therefore, this paper investigates the catalytic performance of 13X zeolite modified with transition metals (such as Fe, Co, Cu) used as a catalyst in the pyrolysis process in a fixed-bed reactor in two stages of the residual rape biomass. The monometallic catalysts such as Fe, Co, and Cu, and bimetallic catalysts such as Fe-Co, Fe-Cu, and Co-Cu modified 13X catalysts were prepared by the wet impregnation method and they were characterized. The aim of this study was to improve the quality of bio-oil produced by residual rape biomass pyrolysis, and to provide details about performance of metal-modified 13X zeolite catalysts used in this pyrolysis process.

## 2. Experimental Part

### 2.1. Materials and Methods

Residual biomass used in this study was rapeseed residue (straw, leaves, and pods) collected from the local area (Figures 1(a) and 1(b)).

The bio-waste was first dried at 105°C until it reaches a constant mass and then ground and sieved through a 60 mesh sieve. The final biomass was labeled as residual rapeseed biomass (RRB). The RRB used was a fraction of ≤60 mesh (of ≤0.25 mm) to minimize the heating and mass transfer impact and to reduce the temperature gradients into the RRB sample. To determine the fixed carbon, moisture, volatile, and ash content, proximate analysis of the RRB was performed according to ASTM standards D 2016 74, D3174 89, and D1102 84. By the ultimate analysis, the content of carbon, hydrogen, nitrogen, and sulfur was determined. The oxygen concentration was calculated by difference till 100%. A Carlo Elba 1106 instrument and ASTM D 5373 standard were used. The rapeseed residual biomass composition was established according to ASTM D 3176 and the ASTM D240-02 was used to determine the gross calorific value (GCV). The extractives and lignocellulosic content of RRB were determined using TAPPI method, as is described in reference [43]. The organic structure of RRB was established by Fourier infrared spectroscopy and an FTIR spectrometer Nicolet iS50 was used. Also, a thermogravimetric analysis of RRB was performed and for this a Setaram Setsys Evolution instrument coupled with a PC was used. The N_2_ of 99.99% purity, at 50 ml/min flow rate, 20°C/min heating rate up to a final temperature of 900°C, and 50 mg of sample mass, were analysis parameters. All tests were repeated three times, and the values represent the average of these three measurements. The data standard deviations are provided and the relative error is less than 1.5%.

### 2.2. Catalysts Preparation

Cobalt nitrate [Co(NO_3_)_2_.6H_2_O], ferric nitrate[Fe(NO_3_)_3_.9H_2_O], and copper nitrate [Cu(NO_3_)_2_.3H_2_O], of analytical grade were purchased from Sigma-Aldrich and used as metal precursors. The 13X zeolite in pellets form (Ɵ = 3 mm), having a Si/Al ratio = 3.2 was purchased from FLUKA of Sigma-Aldrich Holding AG, milled, and sieved through a 60 mesh sieve to obtain the particles with a size ≤0.25 mm. Before being used, the 13X zeolite was calcined at 500°C for 4 hours. Previous studies [44, 45] suggest that a metal loading on catalytic support up to 10 wt.% is the optimum value to create a sufficient number of strongly active states for deoxygenation reaction, and that a higher amount of metal can reduce the number of active states and as a result the catalytic activity is also reduced. Considering this finding, the catalysts were prepared with a metallic load of ≤10 wt.%. Metal-modified 13X zeolite catalysts (M/13X; M = Fe, Co, Cu) were prepared by the wet impregnation technique. First, the amounts of ferric nitrate [Fe(NO_3_)_3_.9H_2_O] (72.14 g), cobalt nitrate [Co(NO_3_)_2_.6H_2_O] (49.33 g), and copper nitrate [Cu(NO_3_)_2_.3H_2_O] (38.05 g), containing 10 g of each metal were calculated. Each of the amounts of these compounds were weighed and dissolved in 100 ml of distilled water. The solution of ferric nitrate [Fe(NO_3_)_3_.9H_2_O] had a concentration of 1.78 mol/L, cobalt nitrate [Co(NO_3_)_2_.6H_2_O] had a concentration of 1.69 mol/L, and copper nitrate [Cu(NO_3_)_2_.3H_2_O] had a concentration of 1.57 mol/L. Then, 100 g of 13X zeolite having particle size of ≤0.25 mm, was impregnated with each 100 ml aqueous solutions of ferric nitrate, cobalt nitrate, and copper nitrate, without stirring, at room temperature for 8 h. The resulted mixtures were dried at 105°C for 12 h, and then the samples were calcined in a furnace at 500°C for 6 h. After cooling, the samples were labeled as Fe/13X, Co/13X, and Cu/13X, respectively. The metal content from each sample was determined by atomic absorption analysis, using a spectrophotometer type Analytic Yena Nova 300 and the content of metal (Fe, Co, and Cu) into 13X zeolite was ∼5.5 wt.%.

The preparation of bimetallic catalysts (Fe-Co/13X, Fe-Cu/13X, and Co-Cu/13X) was performed as follows: Each mixture of ferric nitrate [Fe(NO_3_)_3_.9H_2_O] (72.14 g) + cobalt nitrate [Co(NO_3_)_2_.6H_2_O](49.33 g); ferric nitrate[Fe(NO_3_)_3_.9H_2_O](72.14 g) + copper nitrate [Cu(NO_3_)_2_.3H_2_O] (38.05 g); cobalt nitrate [Co(NO_3_)_2_.6H_2_O] (49.33 g) + copper nitrate [Cu(NO_3_)_2_.3H_2_O] (38.05 g) was added to 100 ml of distilled water at room temperature and stirred (400 rot/min) until it was completely dissolved. After that, samples of 100 g 13X zeolite(particle size ≤0.25 mm) was impregnated with aqueous solutions of Fe-Co, Fe-Cu, and Co-Cu without stirring for 8 h. The resulted mixtures were dried at 105°C for 12 h. Finally, the dried mixtures were calcined at 500°C for 6 h. The resulting catalyst samples were labeled as Fe-Co/13X, Fe-Cu/13X, and Co-Cu/13X. The metal content from each sample was determined by atomic absorption analysis, using a spectrophotometer type Analytic Yena Nova 300 and the content of metal (Fe, Co, and Cu) into 13X zeolite was ∼5.8 wt.%.

### 2.3. Catalysts Characterization

Phase analysis of the catalysts was performed by X-ray diffraction (XRD), using D/max-2200/PC, Rigaku, Japan, and copper KR radiation (40 kV, 20 mA) as the X-ray source. Metal crystallite size was established using the Scherrer equation:

(1) $$\begin{array}{c} d_{\text{crystallite}}=\frac{0.94\lambda }{B.\;\cos\;\theta }, \end{array}$$

where *d*_crystallite_ size was in nm, *B* was full width at half maximum of most intense peak of spectrum (FWHM), *λ* was considered as 1.5405 Å and 2*θ* between 10 and 90 degree.

The energy dispersive X-ray fluorescence (EDXRF) analysis was used to determine the metals from catalyst composition. The N_2_ adsorption/desorption isotherms of the catalysts, at (−196.15°C) were drawn, using Quantachrome Inst., Nova 2200e analyzer, and the Brunauer–Emmett–Teller method was used to establish the specific surface area, the total pore volume was determined at a relative pressure of *P*/*P*_o_ = 0.99, and the pore size distribution resulted from the Brunauer–Joyner–Halenda (BJH) model. Scanning electron microscopy (SEM) was used to analyze the catalysts' morphology (SEM) and a JSM-7500F microscope(JOEL-Japan) was used, operated at 10 kV, using gold coating. The variations of acidity after introducing the metals established ammonia adsorption. A TPD Nuchrom analyzer with a thermal conductivity detector was used to perform the TPD-NH_3_ experiments. NH_3_-TPD experiments were performed on the samples of the catalyst which were preheated for 60 mins at 300°C, then the samples were cooled at 45°C and the catalyst sample was saturated by ammonia gas by passing onto the catalyst reactor at 45°C. After base line restoration, the sample was heated from 45 to 750°C, with a heating rate of 10°C/min in helium flow of 50 mL/min.

### 2.4. Pyrolysis Experimental Test

Catalytic pyrolysis experiments were performed in a fixed-bed reactor in two stages. The scheme of the pyrolysis system is presented in Figure 2. It mainly consists of a biomass feeding unit, an inert gas supplying unit, a fixed-bed reactor in two stages, condensers coupled to the bio-oil collection vessels, a glass wool filter, gas flowmeter, thermocouples for temperature measurement, sampling point, and gas storage tank. The reactor is made of stainless steel with a height of 950 mm and an internal diameter of 52 mm and is divided into the following sections: (i) a section for biomass pyrolysis with a height of 400 mm (stage I); (ii) a catalytic section for pyrolysis vapors with a height of 350 mm (stage II); (iii) a final part of the reactor with a height of 200 mm that is the area for collecting and removing products from the reactor.

The reactor was electrically heated (3) and two thermocouples (5 and 6) were placed in the zone of stage I and zone of stage II to measure the temperature from both areas. In order to ensure an inert atmosphere in the reactor during the pyrolysis process and to help evacuate pyrolysis products, an inert gas (N_2_), at a flow rate of 60 ml/min, was continuously passed through the system. The condensers (8 and 9) were held to 15–20°C by circulating cold water (≈8–10°C) and had the role to cool condensable and noncondensable gas fraction. Final condensation of vapors takes place in the collecting vessels (10 and 11) and the final condenser (14) is cooled with water of 5°C. Prior to each pyrolysis test, 100 g of catalyst was introduced into the reactor in the catalytic zone (stage II), then N_2_ gas, at a flow rate of 60 ml/min was passed through the reactor to evacuate the air. Then, the whole reactor was heated to 500°C with a heating rate of 20°C/min.

When the temperature in the reactor was reached and stabilized, 100 g of residual rapeseed biomass was introduced into the reactor in the pyrolysis zone (stage I). Rapeseed residual biomass placed into the pyrolysis zone adsorbed heat, a thermal degradation took place, and pyrolysis vapors including moisture, condensable, and noncondensable gases and also aerosols were formed, together with a solid residue (bio-char). The pyrolysis vapors passed on and reached the area containing the catalyst bed (stage II) and there were more reactions, such as cracking, deoxygenation (by decarboxylation, decarbonylation, and dehydration), and polymerization which took place, resulting in much more aliphatic and aromatic compounds. The upgraded catalytic pyrolysis vapors passed on glass wool filter (7), where the fine particles were retained, then entered into the condensers (8 and 9) and the condensable volatiles were transformed to liquid which was collected in vessels (10) and (11) where cooling continued. The noncondensable gases were collected and stored in system (16). The samples of noncondensable gases were used to analyze the compositions, and the volume was measured using the gas flowmeter (15). The experimental test took place for 30 min, after this period, no significant release of gas was observed and measured. After the experimental test, the heating of the system was interrupted and N_2_ gas further passed through the system until the reactor cooled to room temperature, thus preventing the oxidation of bio-char. From the pyrolysis zone, the bio-char was collected and by weighing, the bio-char amount was determined. The coke deposited on the catalyst was determined by the weight loss of the spent catalyst, before and after it was burnt with air in an oven for 2 hours, at a temperature of 500°C. The amount of liquid was determined by the difference in weight of the collection vessel (10 and 11) after and before the experiment. The noncondensable gas yield was determined by the overall mass balance.

### 2.5. Characterization of the Catalytic Pyrolysis Products

The chemical bio-oil composition was established by GC-MS analysis (gas chromatography-mass spectrometry method). A GCMS-QP2010SE gas chromatograph/mass spectrometer was used and the identification of chromatographic peaks were performed according to the NIST08 and Wiley mass spectrum library. The relationship between the concentration of each compound and its area given by the corresponding peak in the diagram was used to determine the bio-oil composition. The compositional analysis of the functional groups was carried out by using a Nicolet 6700 FTIR spectrophotometer and using KBr tablets of 1 mm thickness. The density of bio-oil was measured according to ASTM D 1298. The water content from bio-oil was determined by Karl Fischer method, according to ASTM D 1744 and the ash content was according to ASTM D 482. The sulfur content was established according to the IP336 method and the carbon residue according to ASTM D 189. The caloric value was measured according to ASTM D 3286-91a, and total acid value was established according to ASTM D 974. The bio-oil pH value was determined using a digital pH meter (Mettler Delta 340). The empirical formula, H/C, N/C, and O/C molar ratios were established from elemental composition. The bio-oil kinematic viscosity was measured using a ARES TA rheometer, with the temperature being set at 25°C and 60°C. The bio-oil surface tension was measured at 25°C, for this, the Wilhelmy plate method was used.

The composition of gas product was determined by gas-chromatograph analysis for this using a chromatograph type Varian CP-3800 equipped with TCD and FID detectors. The chromatograph was also equipped with the next three columns: (i) a column with a length of 2 m, a diameter of 0.00315 mm that contains 5 Å molecular sieve as filling; (ii) a column with a length of 6 m, a diameter of 0.00317 containing Porapak N, and (iii) a column with a length of 1 m, a diameter of 0.0018 mm, containing Chromosorb. Argon (99.999 vol.%) provided by Linde Company, was used as the reference gas. The concentration of N_2_, CO, CO_2_, H_2_, CH_4_, and hydrocarbons up to C_7_ components were determined. After each experiment, the solid product (bio-char) was collected from the reactor and its quantity was determined by weighing. Each experimental test was repeated three times for the same process conditions. The results represent the average values of these data.

## 3. Results and Discussion

### 3.1. Rapeseed Residual Biomass Characterization

Rapeseed residue (including straw, leaves, and pods, Figure 1) collected from the local area was characterized and the proximate, ultimate, component analysis, and gross caloric value are shown in Table 1. To limit the amount of water that reaches the bio-oil, the moisture content of the raw material (biomass) should be below 10 wt.%. [9, 11]. From the results shown in Table 1, it can be observed that the moisture amount of rapeseed residual biomass is 8.35wt.%, which is under 10wt.% value. The gross caloric value is 19.23 (MJ/kg) and is similar to other agricultural residual biomass (such as sunflower stalks) [46].

The FT-IR spectra of the rapeseed residual biomass is presented in Figure 3.

The (O–H) vibrations for the hydroxyl groups have appeared in the band from 3400 to 3350 cm^−1^. The band above 3500 cm^−1^ could be attributed to unbound O-H groups for phenols, alcohols, or carboxylic acids. The band in the area with a wavelength greater than 3500 cm^−1^ was correlated with the existence of a large number of OH groups with symmetrical and asymmetric stretching vibrations (H_2_O molecules). The band in the range 2925 cm^−1^–1400 cm^−1^ was attributed to the vibration of the C–H, –CH_2_, and –CH_3_ groups, respectively, from the aliphatic chain. These aliphatic chains represent the basic structure of the lignocellulosic biomass [47]. Carboxylic acids and carbonyl groups of esters are shown at the peak of about 1700 cm^−1^, and the peak of about 1530–1600 cm^−1^ is probably due to aromatic hydrocarbons.

The curve of the thermogravimetric analysis is shown in Figure 4(a).

As can be seen in Figure 4(a), the weight loss increased with the increase of temperature. When the pyrolysis of rapeseed residual biomass sample was finished, it yielded a residue of 37.14 wt. %. The DTG curve presents the thermal degradation of the sample (Figure 4(b)). The initial weight loss temperature (Ti) was about 145°C, the temperature after the reaction completed (Tf) was about 620°C, and the maximum weight loss was at the temperature at which the maximum peak appeared (T_peak_) of about 320°C. The DTG curve of rapeseed residual biomass shows a wide peak with a shoulder, this profile of thermal degradation is mostly observed for biomass that is a heterogeneous solid.

The data presented in Table 1 and Figures 3 and 4 show that rapeseed residual biomass represents a suitable raw material source for bio fuel (bio-oil) production by pyrolysis process.

### 3.2. Catalysts Characterization

#### 3.2.1. Metal Content

Metal content in catalysts was determined by atomic absorption analysis. The amount of the introduced metals in modified 13X catalysts is presented in Table 2. For all catalyst samples, the corresponding metal content was in the range 5.45 to 5.87 wt.%, which showed that the impregnated metal amount was almost constant.

#### 3.2.2. Surface Area and Porosity Texture

Specific surface area and porosity texture of 13X zeolite and metal/13X zeolite catalysts were determined and are presented in Table 3.

Compared to the parent 13X zeolite, the specific surface area of the metal-modified catalysts has decreased and in addition, compared to the monometallic catalysts (Fe/13X zeolite, Co/13X zeolite, and Cu/13X zeolite), the specific surface area of the bimetallic catalysts (Fe-Co/13X zeolite, Fe-Cu/13X zeolite, and Co-Cu/13X zeolite), was lower. This results were also presented in other studies [32, 42, 48]. A decreasing trend for pore volume and pore diameter was observed and this is due to the metal species that were distributed on the surface of the 13X zeolite and were even dispersed in the parent zeolite channels. The pore diameter indicates that mainly pore diameter corresponds to mesopores, in the range 2–50 nm which is ascribed to the 13X zeolite used as support. The N_2_ adsorption–desorption isotherms helped us to conclude that the decreasing of surface area and pore volumes of the catalysts are due to impregnation of the porous 13X zeolite support with low surface area metal oxides [49].

#### 3.2.3. XRD and SEM

The XRD patterns of the parent 13X zeolite and the modified 13X zeolite catalysts loaded with Fe, Co, and Cu metals are shown in Figure 5.

A high similarity can be seen between 13X zeolite and mono and bimetallic catalysts (Figures 5(a) and 5(b)). This shows that the 13X zeolite network was preserved even after the metals were loaded into the zeolite mass. Compared to the parent 13X zeolite and monometal-modified catalysts (Fe/13X zeolites, Co/13X zeolites, and Cu/13X zeolites, respectively, Figure 5(a)), the maximum peak intensities after loading with two metals (Fe-Co/13X zeolite, Fe-Cu/13X zeolites, and Cu/13X zeolites, respectively, Figure 5) are diminished.

Monometallic and bimetallic/13X zeolite catalysts were characterized by SEM analysis and in Figure 6 are shown in the SEM images. As can be seen, mono- and bimetallic-modified zeolites catalysts have similar surface morphologies (Figures 6(a)–6(f)).

Figures 6(b)–6(g) show the SEM images of mono and bimetallic catalysts with magnification of 5,000 times, and it can be observed that small particles are distributed on the zeolite surface, without an agglomeration of particles, the morphology of the 13X zeolite has largely not changed by the loading of metal species. Figure 6(a) shows the SEM image of 13X zeolite, and it can be observed that pores are distributed on the 13X zeolite surface and they make possible an easy absorption of the impregnation solution for metal loading.

Moreover, there are no diffraction peaks characteristic of other crystals, except for the typical 13X zeolite peaks, which show that the metals were uniformly dispersed in the zeolite mass and no agglomerations occurred.

#### 3.2.4. Acidic Properties of Catalysts

The strength and quantity of acidic sites present on the surface of the catalysts influence the activity and the performance of the catalysts. The acidity variations of the catalysts produced by the NH_3_-TPD are presented in Figure 7. The acidic strengths of the zeolite-13X support as well as for all metal/zeolite-13X catalysts were established by carrying out the NH_3_-TPD experiments in the range of temperature from 45 to 750°C (Figures 7(a) and 7(b)). The total acidity of the 13X zeolite support and the metal catalysts is given in Table 3. 13X zeolite shows only one wide peak in the range of 100–225°C, whereas two or three wide peaks are shown for all metal/zeolite-13X catalysts: the first peak is shown in the temperature range of 100–240°C, the second one peak is shown in the temperature range of 200–380°C, and the third wide peak is shown in the temperature range of 400–680°C.

The peak situated in the temperature range of 100–225°C shows the ammonia desorbed from the weak acidic sites (physical adsorption of ammonia). The peak in the temperature range of 200–380°C shows the ammonia desorbed from the bronsted sites which are present on the catalyst surface, whereas the wide peak in the high temperature range of 400–680°C shows the ammonia desorbed from the Lewis sites that are present on the catalyst surface. The 13X zeolite contains small amounts of stronger acidic sites in the high temperature range. The increase of acidity for all the metal/zeolite-13X catalysts is due to the impregnation of metal precursors on the 13X zeolite support. It can be observed from Table 3 that the ammonium quantity adsorbed in the bimetallic catalyst is between 7.36 and 9.21 mmol/g which is bigger than that adsorbed in monometallic catalysts (6.24 to 6.84 mmol/g). The overall results (Table 3) show that the catalysts obtained by impregnation have more total acidic sites than that of 13X zeolite. The desorbed quantity of ammonia from one gram of material is associated with material acidity and the order was Cu > Co > Fe > 13X zeolite for monometallic catalysts and Fe-Cu > Fe-Co > Co-Cu > 13X zeolite for bimetallic catalysts.

### 3.3. Distribution of the Products Resulted from RRB Pyrolysis

As mentioned, the distribution of the products can be influenced by several factors, including the presence or absence of the catalyst in the pyrolysis process.  Figure 8 shows the product distribution resulting from the experiments performed in this study with and without the use of a catalyst and the influence of the 13X zeolite and metal-modified 13X zeolite catalysts on this product distribution. The liquid fraction which resulted as the product was further separated into aqueous phase and bio-oil phase. The catalytic tests were performed under the same operating parameters with and without catalyst. Furthermore, the parent 13X zeolite was used in order to compare the effect of metal introduction into 13X zeolite mass. The addition of 13X zeolite in the pyrolysis process decreased the liquid fraction which consists of bio-oil and aqueous phases, from 47.38.% to 43.15 wt.%, while the gas fraction increased from 24.85 wt.% to 31.25 wt.% against without catalyst pyrolysis process, as can be seen in Figure 8. During the catalytic pyrolysis process, biomass also goes through a series of stages of thermal decomposition (such as dehydration, decarbonylation, and decarboxylation) resulting in cracking reactions and releasing of volatiles as noncondensable gases [16, 18].

Moreover, the addition of metals to 13X zeolite had, as result, a decrease of bio-oil fraction as compared to the use of parent 13X zeolite (i.e., from 13.65 wt.% for 13X zeolite to 7.85 wt.% for Fe/13X zeolite, respectively), which could be attributed to a pronounced dehydration process that took place and was favored by metal-modified 13X zeolite catalysts [44]. Regarding the variation of acidity of the catalysts, an increase of the acidity was observed for the modified metal 13X zeolite catalysts compared to the parent 13X zeolite (Table 8). Compared to the treatment with Fe and Co/13X zeolite catalysts, the introduction of Cu improved the bio-oil fraction and gas phase. The highest amount of bio-oil fraction (12.56 wt.%) and gas phase (31.52 wt.%) were obtained by the Fe-Cu/13X zeolite catalyst. Moreover, the quantity of solid fraction (char and coke) has generally remained unchanged (in the range 24.53–25.73 wt.%), indicating a high consistency of the pyrolysis process for each test at the constant pyrolysis temperature (500°C), the almost same metal loading rate (5.45 wt.% to 5.85 wt.%, see Table 2) on the parent 13X zeolite, and the constant biomass/catalyst ratio (1 : 1).

### 3.4. Products Distribution in the Bio-Oil Phase

The composition of the bio-oil resulted on different metal/13X zeolite catalysts shown in Figure 9. Compared to the experiment performed without catalyst, addition of 13X zeolite as catalyst decreased the undesired compounds containing oxygen, from 62.45% to 21.38%, and the selectivity to aromatics products was improved. This behavior is attributed to the presence of acidic sites onto 13X zeolite which catalyzed the deoxygenation reactions through dehydration, decarbonylation, and decarboxylation, followed by the reactions of cyclization and aromatization [16, 32, 50]. In the case of monometallic catalysts, the content of oxygenated compounds was substantially reduced from 62.45% to 31.07% for Cu/13X zeolite, 28.05% for Co/13X zeolite, and 25.41% for Fe/13X zeolite, respectively.

This behavior is probably due to the combining effects of the acidic sites strength and metal sites during catalytic conversion reactions. In the case of bimetallic catalysts, a higher selectivity was observed for the aromatization reactions, resulting in higher amounts of aromatic hydrocarbons in bio-oil composition as follows: 31.85% for Fe-Co/13X zeolite, 33.18% for Co-Cu/13X zeolite, and 35.28% for Fe-Cu/13X zeolite, respectively, compared with 25.32% for 13X zeolite. It can be observed that, compared to the pyrolysis without catalyst, the content of phenols in the bio-oil produced with catalysts is significantly increased. Among all the monometallic-modified 13X zeolite, the presence of Fe/13X zeolite during catalytic pyrolysis behaved the best, and the phenols content increased from 13.25% to 35.05%. The content of phenols reached the highest value of 34.72% over the bimetallic catalyst Fe-Co/13X zeolite. This is mainly due to the increased production of light compounds with smaller molecules that resulted from the catalytic cracking of pyrolysis vapors [42]. Compared to the experiment without catalyst and the parent 13X zeolite, it was observed that the aliphatic content in oil composition has increased in the presence of Co/13X zeolite catalyst, but after loading with Fe and Cu of the 13X zeolite, the aliphatic content decreased. This behavior could be explained by the fact that loading with Fe and Cu would favor the aromatization reactions of aliphatic hydrocarbons, as shown in other studies [46, 51, 52]. In addition, the content of compounds containing nitrogen into the bio-oil composition was significantly decreased compared to the experiment without catalyst, this being mainly due to the presence of acidic and metallic states in the structure of catalysts, which are considered to favor decomposition and aromatization reactions, and nitrogen-containing compounds are transformed into aromatic compounds [18, 28].

#### 3.4.1. Aromatic Hydrocarbons Distribution in Bio-Oil

Aromatic hydrocarbons can be divided in monocyclic aromatic hydrocarbons (MAHs) including benzene, toluene, ethylbenzene, and xylene, and polycyclic aromatic hydrocarbons (PAHs) which include compounds such as naphthalene, anthracene, and phenanthrene. The polycyclic aromatic hydrocarbons cause coke formation on the catalyst surface leading to the catalyst deactivation [2].  Figure 10 shows the influence of catalysts on the selectivity for aromatics distribution (MAHs and PAHs) in the bio-oil composition. It can be seen that metal/13X zeolite catalysts showed higher selectivity for MAHs compared to the experiment without catalyst and in the presence of 13X zeolites.

The MAHs content increased from 1.05 (experiment without catalyst) to 12.65% (experiment using 13X zeolite) and to 14.18–27.45% (experiment with mono and bimetallic 13X zeolite catalysts), respectively. It is assumed that this behavior is due to the combination of the effects of acid sites and metal sites of metal catalysts [16, 18]. The organic compounds from bio-oil composition were activated and cracked, and a part of APHs was possibly converted to MAHs[32, 53]. In the presence of different metal/13X zeolite catalysts, the selectivity to MAHs was improved with varying degrees. In the experiment performed in the presence of Fe-Cu/13X zeolite catalyst, the MAHs content was above 27.45%, followed by Co-Cu/13X zeolite catalyst with 22.68% and Fe-Co/13X zeolite catalyst with 20.35%, respectively, this indicating that the bimetallic 13X zeolite catalysts are suitable to be used to convert the biomass pyrolysis vapors to fuels containing mainly light hydrocarbons.

#### 3.4.2. Oxygenated Compounds Distribution in Bio-Oil

The effects of the metals/13X zeolite catalysts on the distribution of oxygenated compounds in the bio-oil are shown in Figure 11. Several types of oxygenated compounds have been identified in the composition of the bio-oil, including mainly aldehydes, alcohols, ketones, acids, esters, furans and other organic compounds. Among them, aldehydes, acids, and ketones showed a strong reactivity due to the presence of the carbonyl group (C=O), which proved to be the main cause of the instability and degradation of the bio-oil. Although alcohols and furan have a relatively high stability and added value, the oxygen in their composition does not cause an improvement in the calorific value of the bio-oil. It is therefore necessary to reduce as much as possible the amount of the various oxygenated compounds in the bio-oil and to convert them to hydrocarbons.

Oxygen can be removed in the form of H_2_O, CO, and CO_2_ mainly by dehydroxylation (R-OH⟶R1 + H_2_O), decarbonylation (R-COH⟶R-H + CO), and decarboxylation (R-COOH⟶R-H + CO_2_) reactions. As can be seen in Figure 11, the content of oxygenated compounds decreased significantly in the composition of the bio-oil resulting from pyrolysis in the presence of catalysts, compared to the situation without catalyst. Furthermore, bimetallic catalysts were more efficient in removing oxygenated compounds compared to parent 13X zeolites and monometallic catalysts. As can be observed from Figure 9, the total amount of oxygenated compounds decreased from 62.45 wt.% (without catalyst) to 16.05 wt.% in the presence of Co-Cu/13X zeolite catalyst. On the other hand, as shown in Figure 11, the best behavior had the Fe-Cu/13X zeolite catalyst, the aldehydes, alcohols, acids, and esters were almost completely removed, while the ketone content was reduced from 28.67 wt.% to 11.07 wt%, compared to the situation without catalyst. In addition, the furan content increased from 1.35 wt.% for the situation without catalyst to 10.26 wt.% in the case of Fe-Cu/13X zeolite catalyst. This means that during the deoxygenation reaction, amounts of oxygen-containing carbocations were cyclized and converted to furan. The presence of Fe-Cu/13X zeolite catalyst effectively decreased the content of carbonyl compounds which affected the bio-oil stability to a much smaller value and significantly increased the content of desired components, so the quality of bio-oil was effectively improved. Among all the catalysts used in this study, Fe-Cu/13X zeolite catalyst showed a higher performance for improving the quality of rapeseed biomass pyrolysis bio-oil.

### 3.5. Characteristics of Bio-Oil Obtained by Rapeseed Residual Biomass Pyrolysis

The pyrolysis experiments showed that the catalyst Fe-Cu/13X zeolite catalyst performed best in improving the bio-oil quality. Analyses were performed to determine the physico-chemical properties of the bio-oil, and the results are shown in Table 4. It can be clearly seen that 13X zeolite reduced the oxygen content from 31.98% by weight to 23.22% by weight, while Fe-Cu/13X zeolite catalyst reduced it to 16.06% by weight. This shows that the 13X zeolite and Fe-Cu/13X zeolite catalysts performed well in the deoxygenation process and improved the quality of the bio-oil. In addition, bio-oil obtained from the pyrolysis of rapeseed residual biomass has a lower sulfur content compared to light and heavy commercial fuel. This could be an important advantage for the use of biomass resources, as it can reduce the emission of sulfur compounds, mitigating environmental pollution.

Further, a decreasing of nitrogen content was observed which could be due to the denitrification reaction under the catalytic pyrolysis conditions [31]. Also, a decreasing of H/C molar ratios was observed of the bio-oil resulted from the catalytic experiments than in the bio-oil obtained from pyrolysis without catalyst, which would indicate an increasing in aromatic compounds and a decreasing in aliphatic products. The decrease of the O/C molar ratios of the bio-oil obtained from catalytic experiments also showed a high deoxygenation effect of 13X zeolite and Fe-Cu/13X zeolite catalysts. As a result, an improvement in GCV for bio-oil obtained from catalytic pyrolysis was observed. The GCV of 33.85 MJ/kg was for bio-oil obtained by Fe-Cu/13X zeolite catalyst which showed the best performance, also the viscosity for the same bio-oil decreased to 45.17 mm^2^/s (Table 4), this meaning an improvement of bio-oil flow characteristics. As can be seen in Table 4, an increase of the pH value was obtained for the bio-oil produced from catalytic experiments, indicating that acids content was reduced; this being a proof of improvement of the bio-oil characteristics, the corrosion effect being also reduced. Moreover, the bio-oil density decreased slightly, which increased the atomization effect of the fuel. However, the values of pH, density, and viscosity, still must be improved, there is a definite difference to the quality of the commercial light and heavy fuel oil, as can be seen in Table 4. On the other hand, the results obtained in this study show a good behavior and high performance of 13X zeolite modified with transition metals in the biomass vapors pyrolysis process, these being similar to those obtained, for example, with catalysts based on ZSM-5 [18, 29].

### 3.6. Gaseous Fraction Composition

Table 5 presented the gas composition resulted from the pyrolysis of rapeseed residual biomass without catalyst and in the presence of metals/13X zeolite catalysts.

As can be observed, the usage of metals/13X zeolite catalysts increased the CO_2_ content compared to the pyrolysis in the presence of parent 13X zeolite, this means the modified 13X zeolite catalysts improved the decarboxylation reaction, resulting in the form of CO_2_ emission. Moreover, using metal catalysts promoted the H_2_ generation, and the highest H_2_ content of 9.38% was obtained with the Fe/13X zeolite catalyst. This could be due to the dehydrogenation of the aliphatic hydrocarbons to olefins and then during the aromatization of the olefins to aromatics hydrocarbons. As can be seen, monometallic catalysts performed higher CH_4_ content compared to bimetallic catalysts, in fact when Fe-Co/13X zeolite, Fe-Cu/13X zeolite, and Co-Cu/13X zeolite catalysts were used, the CH_4_ amount decreased, this could be attributed to the CH_4_ aromatization process [31]. Also, the content of C_2_-C_7_ aliphatic hydrocarbons decreased in the presence of bimetallic catalysts compared to the use of monometallic catalysts. This behavior could be explained as follows, when hydrocarbons C_2_-C_7_ co-reacted with CH_4_, the C_2_-C_7_ hydrocarbons became active to dehydrogenation reactions and their transformation into olefins, while CH_4_ was activated by the reaction of hydrogen transfer between CH_4_ and olefins, resulting in enhanced aromatization of CH_4_ [29]. As a result, the aromatics content was the highest when Fe-Cu/13X zeolite was used, being 35.28% as can be seen in Figure 9. The catalyst based on the combination of Fe and Cu presented the best behavior in aromatization process of pyrolysis vapors.

## 4. Conclusions

In this study, the 13X zeolite was modified with transition metals (M = Fe, Co, Cu) and mono and bimetallic catalysts were prepared. This catalysts were used for rapeseed residual biomass pyrolysis in a two-stage system to produce bio-oil. The loading rate of the metal in the zeolite mass was relatively constant (ranging from 5.45 to 5.87 wt.% on parent 13X zeolites), pyrolysis for each test was performed at a constant temperature (500°C) and the biomass/catalyst ratio was maintained constant (1 : 1). The content of oxygenated compounds decreased significantly in the composition of the bio-oil resulting from pyrolysis in the presence of catalysts, compared to the situation without catalyst. The most efficient catalyst proved to be Fe-Cu/13X zeolite, which exhibited high selectivity for MAHs (27.45%) and a deoxygenation performance from 62.45% to 20.56%. The decrease of the O/C molar ratios in the bio-oil obtained from catalytic experiments showed a high deoxygenation effect of mono and bimetallic/13X zeolite catalysts and as a result, an improvement in GCV for bio-oil was observed. Also, the viscosity for the obtained bio-oil decreased, this meaning an improvement of bio-oil flow characteristics. The increase of the pH value for the bio-oil produced from catalytic experiments, indicated that the content of acids was reduced; this being a proof of improvement of the bio-oil characteristics, the corrosion effect being also reduced. On the other hand, the monometallic catalysts performed higher CH_4_ content compared to bimetallic catalysts. The catalyst based on the combination of Fe and Cu presented the best behavior in the aromatization process of pyrolysis vapors. The obtained results show that by modifying the 13X zeolite with transition metals such as Fe, Co, and Cu, catalysts with good performances in the pyrolysis process can be obtained for application in the production of bio-oil with improved properties.

## Figures and Tables

**Figure 1:** Rapeseed residual biomass: (a) straw, leaves, and pods; (b) residual rapeseed biomass ground and sieved to the particle size of ≤0.25 mm.

**Figure 2:** Scheme of experimental setup for biomass pyrolysis. (1) tank with N_2_ gas under pressure; (2) reactor; (3) electrical furnace; (4) biomass feeding; (5) and (6) thermocouples for temperature control; (7) glass wool filter; (8) and (9) heat exchangers for cooling and condensing vapors; (10) and (11) gas-liquid separator containing liquid product; (12) and (13) cooling bath with water (5°C); (14) final condenser with water (5°C); (15) flowmeter; (16) system for gas product including collector (C) and storage tank (T); (V) valve; (IP) pressure indicator; (GC) gas analyzer.

**Figure 3:** FT-IR spectrum of rapeseed residual biomass.

**Figure 4:** TG curve of rapeseed residual biomass (a) and DTG curve of rapeseed residual biomass (b).

**Figure 5:** XRD patterns of; (a) 13X zeolite and monometal/13X zeolite catalysts and (b) 13X zeolite and bimetal/13X zeolite catalysts.

**Figure 6:** SEM images of catalysts and 13X zeolite: (a) 13X zeolite; (b) Fe/13X zeolite; (c) Co/13X zeolite; (d) Cu/13X zeolite; (e) Fe-Co/13X zeolite; (f) Fe-Cu/13X zeolite; (g) Co-Cu/13X zeolite; 30 kV x 5000.

**Figure 7:** TPD-NH_3_ profiles of (a): 13X zeolite; Fe/13X zeolite; Co/13X zeolite; Cu/13X zeolite; and (b): 13X zeolite Fe-Co/13X zeolite; (f) Fe-Cu/13X zeolite; (g) Co-Cu/13X zeolite.

**Figure 8:** Effect of the metal-modified 13X zeolite catalysts on the distribution of products resulted by RRB pyrolysis.

**Figure 9:** Effect of the metal-modified 13X zeolite catalysts on the distribution of compounds in the bio-oil composition obtained by RRB pyrolysis.

**Figure 10:** Effects of the metals/13X zeolite catalysts on the distribution of MAHs and PAHs compounds in the bio-oil composition obtained by RRB pyrolysis.

**Figure 11:** Effects of the metals/13X zeolite catalysts on the distribution of oxygenated compounds in the bio-oil composition obtained by RRB pyrolysis.

**Table 1:** Proximate, ultimate, and component analysis of rapeseed residual biomass (RRB).

Characteristics	RRB
Proximate analysis (wt.%, db)	
Moisture	8.35 ± 0.11
Volatile matter	70.02 ± 1.35
Fixed carbon	15.45 ± 0.25
Ash content	6.18 ± 0.22

*Ultimate analysis (wt.%, db)*	
Carbon	42.05 ± 0.21
Hydrogen	5.12 ± 0.25
Nitrogen	4.18 ± 003
Sulfur	0.71 ± 0.01
Oxygen	47.94 ± 0.25
H/C molar ratio	1.461
O/C molar ratio	0.86

*Component analysis (wt.%, db)*	
Cellulose	47.25 ± 0.2
Hemicellulose	16.45 ± 0.2
Lignin	27.45 ± 0.2
Alcohol/benzene extractives	8.85 ± 0.2
Empirical formula	CH_1.461_ O_0.855_ N_0.085_ S_0.006_
pH	5.57
^b^GCVc (MJ/kg)	19.23

Db: dry basis; ^a^calculated from difference; ^b^gross calorific value.

**Table 2:** Metal content in different metal/13X zeolite catalyst samples.

Catalyst	Fe (wt.%)	Co (wt.%)	Cu (wt.%)
Fe/13X	5.52 ± 0.05	—	—
Co/13X	—	5.45 ± 0.05	—
Cu/13X	—	—	5.55 ± 0.04
Fe-Co/13X	5.75 ± 0.05	5.87 ± 0.06	—
Fe-Cu/13X	5.82 ± 0.04	—	5.76 ± 0.05
Co-Cu/13X	—	5.84 ± 0.03	5.85 ± 0.03

**Table 3:** Surface area (*S*_BET_), pore volume (*V*_p_), pore diameter (*d*_p_), and acidity of 13X zeolite and metal-modified 13X zeolite catalysts.

Catalyst	S_BET_ (m^2^/g)	Pore volume (cm^3^/g)	Pore diameter (nm)	Total acidity_TPD-NH3_ (mmol/g)
13X zeolite	620 ± 2.25	0.434 ± 0.02	11.95 ± 0.15	4.75 ± 0.05
Fe/13X	327 ± 2.05	0.254 ± 0.02	11.12 ± 0.12	6.24 ± 0.05
Co/13X	435 ± 2.21	0.268 ± 0.08	10.35 ± 0.11	6.75 ± 0.05
Cu/13X	468 ± 0.95	0.278 ± 0.04	10.72 ± 0.09	6.84 ± 0.05
Fe-Co/13X	308 ± 2.15	0.255 ± 0.07	11.25 ± 0.15	8.85 ± 0.05
Fe-Cu/13X	303 ± 1.25	0.234 ± 0.05	10.64 ± 0.05	9.21 ± 0.05
Co-Cu/13X	301 ± 1.85	0.262 ± 0.25	10.72 ± 0.35	7.36 ± 0.05

**Table 4:** Characteristics of bio-oils obtained without catalyst and by using 13X zeolite and Fe-Cu/13X zeolite catalysts.

Characteristics	Bio-oil			Commercial crude oil [54]	
	Sample 1	Sample 2	Sample 3	Light crude oil	Heavy crude oil
Ultimate analysis					
C	55.62	68.79	75.42	86.42	88.26
H	768	7.27	7.85	13.35	9.47
N	0.71	0.67	0.61	0.0	0.35
S	0.04	0.04	0.05	0.16	1.55
O^a^	31.98	23.22	16.06	0.07	0.37
H/C molar ratio	1.65	1.27	1.25	1.85	1.29
O/C molar ratio	0.43	0.25	0.16	0.0006	0.003
Viscosity at 50°C (mm^2^/s)	51.26	47.75	45.17	2.00	50.14
pH	5.42	6.05	6.25	0.0	0.0
Density (g/mL)	1.07	1.02	0.97	0.82–0.86	0.83–0.95
GCV^b^ (MJ/kg)	23.65	28.46	33.85	46.0	40.3

Note: Sample 1, the bio-oil obtained without catalyst; Sample 2, the bio-oil obtained using 13X zeolite as catalyst; Sample 3, the bio-oil obtaining using Fe-Cu/13X zeolite as catalyst; a, calculated from difference; b, gross calorific value.

**Table 5:** Influence of metal-modified 13X zeolite catalysts on the gas composition.

Catalyst	1	2	3	4	5	6	7	8
Gas component								
CO	37.65	40.95	28.05	31.42	30.88	42.82	37.12	42.16
CO_2_	52.63	38.78	52.11	49.74	49.95	49.12	53.65	51.76
H_2_	0.85	1.49	9.38	7.63	7.81	4.03	5.96	3.45
CH_4_	5.62	7.15	5.48	5.97	6.01	0.52	0.43	0.29
C_2_-H_7_	3.25	11.63	4.98	5.24	5.35	3.51	2.84	2.34

1, Without catalyst; 2, 13X zeolite; 3, Fe/13X zeolite; 4, Co/13X zeolite; 5, Cu/13X zeolite; 6, Fe-Co/13X zeolite; 7, Fe-Cu/13X zeolite; 8, Co-Cu/13X zeolite.

## Data Availability

The data used to support the findings of this study are included in the paper. Further information or data are available from the corresponding author upon request.
